The article "The circular RNA 001971/miR-29c-3p axis modulates colorectal cancer growth, metastasis, and angiogenesis through VEGFA" was retracted in 2022. Reason: lack of ethics approval or compliance.

# The circular RNA 001971/miR-29c-3p axis modulates colorectal cancer growth, metastasis, and angiogenesis through VEGFA

**DOI:** 10.1186/s13046-020-01594-y

**Published:** 2020-05-19

**Authors:** Chen Chen, Zhiguo Huang, Xiaoye Mo, Yanmin Song, Xiangmin Li, Xiaogang Li, Mu Zhang

**Affiliations:** 1 Department of Pediatrics, Xiangya Hospital, Central South University, Changsha, Hunan People’s Republic of China; 2 Department of Emergency, Xiangya Hospital, Central South University, Changsha, Hunan People’s Republic of China

**Keywords:** Colorectal cancer (CRC), Metastasis, Angiogenesis, Circ-001971, miR-29c-3p

## Abstract

**Background:**

Colorectal cancer (CRC) is one of the most common malignant tumors globally. Angiogenesis is a key event maintaining tumor cell survival and aggressiveness. The expression of vascular endothelial growth factor A (VEGFA), one of the most significant tumor cell-secreted proangiogenic factors, is frequently upregulated in CRC.

**Methods:**

The MTT assay was used to detect the viability of CRC cells. Transwell assays were performed to detect the invasion capacity of target cells. Relative protein levels were determined by immunoblotting. Pathological characteristics of tissues were detected by H&E staining and immunohistochemical (IHC) staining. A RIP assay was conducted to validate the predicted binding between genes.

**Results:**

We observed that circ-001971 expression was dramatically increased in CRC tissue samples and cells. Circ-001971 knockdown suppressed the capacity of CRC cells to proliferate and invade and HUVEC tube formation in vitro, as well as tumor growth in mice bearing SW620 cell-derived tumors in vivo. The expression of circ-001971 and VEGFA was dramatically increased whereas the expression of miR-29c-3p was reduced in tumor tissue samples. Circ-001971 relieved miR-29c-3p-induced inhibition of VEGFA by acting as a ceRNA, thereby aggravating the proliferation, invasion and angiogenesis of CRC. Consistent with the above findings, the expression of VEGFA was increased, whereas the expression of miR-29c-3p was decreased in tumor tissue samples. miR-29c-3p had a negative correlation with both circ-001971 and VEGFA, while circ-001971 was positively correlated with VEGFA.

**Conclusions:**

In conclusion, the circ-001971/miR-29c-3p axis modulated CRC cell proliferation, invasion, and angiogenesis by targeting VEGFA.

## Background

Colorectal cancer (CRC) is one of the most common malignant tumors globally [1]. Despite the use of surgery, the risk of recurrence and cancer-related death in patients with colon cancer remains high [2, 3]. However, even among those who undergo complete resection, the rates of relapse and local or metastatic recurrence in CRC remain high, with metastatic diseases occurring in approximately half of the affected patients during cancer progression [4]. With this background in mind, angiogenesis is increasingly considered a critical process in the development of solid tumors, since angiogenesis can support tumor growth and a mechanism for malignant cells to metastasize from the primary tumor site to distant organs.

The article "The circular RNA 001971/miR-29c-3p axis modulates colorectal cancer growth, metastasis, and angiogenesis through VEGFA" was retracted in 2022. Reason: lack of ethics approval or compliance.

Angiogenesis is a process of vascular remodeling, that is characterized by neovascularization from an existing blood vessel. Angiogenesis widely occurs in the process of fetal development, menstrual cycle and wound closure. In addition, angiogenesis can be found in numerous pathological processes, such as the development of most solid tumors [5], and acts as a critical factor in carcinogenesis [6]. The vascular system that supplies tumor cells serves as an essential factor for the development, growth and metastasis of tumors. As far back as 1963, it was reported that the size of tumors transplanted into isolated perfused organs did not exceed several millimeters [7]. Nevertheless, the tumors transplanted into mice could quickly grow to more than 1 cm^3^ and eventually kill their hosts [8]. Within isolated perfused organs the tumors did not become vascularized, but they did in mice [9]. Thus, in advanced stages of tumor growth, a more efficient vascular system is needed to provide nutrients and to clear metabolites. In fact, within tumor-related practices, inhibition of angiogenesis, primarily by blocking the VEGF (vascular endothelial growth factor) family and the corresponding receptors, has been strongly confirmed to confer clinical benefits, and to prolong the overall survival of treated patients with specific types of diseases, including CRC [6].

The VEGF family and the corresponding receptors play a critical role in microangiogenesis, and can be considered to have prognostic significance for virtually every type of tumor. The VEGF family and the corresponding receptors, the most important angiogenic regulators, frequently show overexpression in metastatic CRC and are directly related to the tumor vascularization degree, tumor growth and the poor prognosis of patients [10]. Among all VEGF family members, VEGFA (vascular endothelial growth factor A) is regarded as one of the most significant tumor cell-secreted proangiogenic factors [11, 12]. The potential of blood VEGFA levels as a predictive biomarker was evaluated in studies involving the efficacy of the antiangiogenic drug cediranib in metastatic CRC, and the neovascularization involved in VEGFA signaling is considered to be a critical mediator of the factor for the angiogenesis, invasion and spread of tumors [13]. High baseline VEGFA levels correlate with poorer progression-free and overall survival [14] and enhanced malignant tumor spread [15, 16]. Bevacizumab is a potent humanized monoclonal antibody to VEGF that, when combined with standard chemotherapy, results in an overall survival of approximately 24 months compared to approximately 20 months for standard chemotherapy alone [13, 17]. Recent reports have revealed that several miRNAs targeting by VEGFA, such as miR-203 [18], miR-497 [19], miR-26a [20], and miR-199a-5p [21], have antitumor effects. Thus, further investigation of the mechanism of abnormal upregulation of VEGFA in CRC might provide novel strategies for metastatic CRC treatment.

The article "The circular RNA 001971/miR-29c-3p axis modulates colorectal cancer growth, metastasis, and angiogenesis through VEGFA" was retracted in 2022. Reason: lack of ethics approval or compliance.

According to the latest high-throughput studies on the human transcriptome, approximately 85 % of the human genome can be transcribed dynamically and generally mostly as non-coding RNAs (ncRNAs) [22–24]. During the past ten years, many observations have reasonably proposed that ncRNAs remarkably participate in complex molecular signaling, which is necessary for structural and functional regulation in various cells and development environments [25]. Therefore, active dysregulation of ncRNAs has been regarded as a crucial factor in the initiation and progression of different pathological conditions [26, 27]. The basal expression of circular RNAs (circRNAs), a new class in the ncRNA network, has been detected in human cells and has a strong impact on the posttranscriptional regulation of gene expression [28, 29]. Unlike the other two types of ncRNAs, long noncoding RNAs (lncRNAs) and microRNAs (miRNAs), circRNAs have covalently linked ends [30]. Gene expression is regulated by some a number of circRNAs that act as ceRNAs (competing endogenous RNAs) [31], also recognized as sponges for miRNAs, to affect the activity of miRNAs [32, 33]. CircRNAs prevent miRNAs from regulating of their target genes [34, 35]. Through further studies on circRNAs, we can provide an in-depth understanding of pathological mechanisms and more effective prevention and diagnosis of the related diseases.

In the present study, previously reported upregulated circRNAs were selected and analyzed to identify circRNAs that may modulate CRC invasion and angiogenesis. Then, the effects of circ-001971 on the capacity of CRC cells to proliferate and to invade on HUVEC tube formation and tumor growth in mice bearing SW620 cell-derived tumors were examined. Next, miRNAs that may target circ-001971 and VEGFA were selected and verified. The dynamic effect of circ-001971/miR-29c-3p on CRC invasion and angiogenesis was examined. Finally, circ-001971, miR-29c-3p, and VEGFA expression and correlation in tissue specimens were determined. Overall, we aimed to provide a new mechanism by which the circ-001971/miR-29c-3p/VEGFA axis modulates CRC invasion and angiogenesis.

The article "The circular RNA 001971/miR-29c-3p axis modulates colorectal cancer growth, metastasis, and angiogenesis through VEGFA" was retracted in 2022. Reason: lack of ethics approval or compliance.

## Materials and methods

### Clinical specimens, cell lines and cell culture

The present study was approved by Xiangya Hospital, Central South University. Colorectal cancer (T) and matched non-cancerous tissues (N) were obtained from 70 CRC patients who underwent primary surgical resection at Xiangya Hospital with written consent and stored at − 80 °C until further use. All clinicopathologic features of the patients are listed in Tables 1 and 2.

**Table 1:** Correlation of the expression of circ-001971 with clinicopathologic features

Clinic-pathological parameters	circ-001971 expression		p
	High	Low	
Gender			
female	20	21	0.808
male	15	14	
Age			
< 50	21	15	0.151
≥ 50	14	20	
Tumorlocation			
Left	10	14	0.435
Rectum	15	15	
Right	10	6	
TNM			
I	2	11	< 0.001
II	5	17	
III	23	5	
IV	5	2	
Differentiation			
Low	21	15	0.151
Moderat and High	14	20	
Tumor size			
< 5	17	22	0.229
≥ 5	18	13	
Lymph node metastasis			
N0	6	30	< 0.001
N1	18	2	
N2	11	3

**Table 2:** Univariate and multivariate analysis for factors related to overall survival using the COX proportional hazard model

Variable	Univariate analysis			Multivariate analysis		
	***p***-value	HR	95%CI	***p***-value	HR	95%CI
Gender						
Female	0.632	0.840	0.411–1.716			
Male						
Age						
< 50	0.926	1.034	0.511–2.092			
≥ 50						
Tumorlocation						
	0.661					
Left	0.642	1.247	0.491–3.170			
Rectum	0.753	0.861	0.339–2.188			
Right						
TNM						
I	0.000			0.000		
II	0.000	0.011	0.002–0.082	0.000	0.008	0.001–0.097
III	0.000	0.022	0.004–0.111	0.000	0.012	0.001–0.138
IV	0.000	0.070	0.016–0.306	0.000	0.047	0.011–0.212
Differentiation						
Low	0.231	1.547	0.757–3.162			
Moderat and High						
Tumor size						
< 5	0.606	0.831	0.410–1.681			
≥ 5						
Lymph node metastasis						
	0.001			0.480		
N0	0.005	0.255	0.098–0.663	0.227	3.552	0.454–27.791
N1	0.718	1.174	0.492–2.801	0.667	1.217	0.497–2.978
N2						
circ-001971						
High						
Low	0.000	6.785	2.764–16.654	0.001	6.456	2.060–20.232

The normal colon epithelial cell line FHC was purchased from ATCC (Manassas, VA, USA). Five CRC cell lines, HT29, HCT116, LoVo, SW480 and SW620, were characterized in detail and were provided by ATCC. Cell lines were cultured in Dulbecco’s modified Eagle medium (DMEM) supplemented with 10% fetal bovine serum (FBS) in a humidified incubator under 5% CO_2_ at 37 °C.

### H&E staining and immunohistochemical (IHC) staining

The tissue samples were excised, washed with PBS, arrested in diastole with 10% potassium chloride solution, weighed, placed in 10% formalin, and embedded in paraffin. Several sections (4–5 mm thick) were prepared, stained with hematoxylin and eosin (H&E) for histopathology by standard procedures and then visualized by light microscopy. For IHC staining, the content of VEGFA was detected by IHC following the previously described method [36]. After deparaffinization, hydration and blockage of endogenous peroxidase, the sections were incubated for 20 min with 10% nonfat milk in PBS in order to block specific sites and then were incubated at 4 °C overnight with primary anti-VEGFA antibody (ab1316, abcam, USA). Then, sections were washed and incubated with HRP-conjugated goat anti-mouse secondary antibody (SV-0004, Boster, China) for 30 min at 37 °C. Finally, the sections were washed and incubated with a DAB kit (AR1022, Boster) for 10 min.

The article "The circular RNA 001971/miR-29c-3p axis modulates colorectal cancer growth, metastasis, and angiogenesis through VEGFA" was retracted in 2022. Reason: lack of ethics approval or compliance.

### Cell viability determined by the MTT assay

The MTT assay was used to detect the viability of CRC cells. Cells were cultured in 96-well plates (5 ×  10^4^ cells/well). Twenty-four hours after plating the cells were attached, and 10 μL MTT was added to the fresh medium to replace the old medium. Four hours after incubation with the medium containing MTT at 37 °C, the medium was discarded, and DMSO (100 μL) was added to each well after discarding the medium. After that, the absorbance was measured at 490 nm. The results are presented as percentage inhibition compared to the untreated control.

### DNA synthesis assays

The ability to synthesize DNA was detected by 5-ethynyl-2′-deoxyuridine (EdU) assays using an EdU assay kit (Guangzhou RiboBio Co., Ltd.) according to the manufacturer’s instructions. Briefly, cells were incubated with EdU for 24 and 48 h in the dark. Then, the cells were fixed with 4% paraformaldehyde for 30 min and stained with Apollo 567 solution for 30 min at room temperature in the dark. The inflorescence absorbance value of each well was determined by a multifunction microplate reader (Bio-Rad, USA).

### Tube formation

The human umbilical vein endothelial cell line HUVEC was purchased from ATCC and seeded in 24-well plates coated with Matrigel (90 μL), incubated at 37 °C for 30 min to polymerize, and then seeded in wells under different SW620 cell-conditioned media (CM) as described. The 24-well plates were incubated for 6 h, and tube formation was then imaged under an inverted microscope at a × 200 magnification.

### Transwell invasion assay

Transwell assays were performed to detect the invasion capacity of target cells. Cells (5 × 10^5^) were plated on the upper chamber of a polycarbonate Transwell filter (Cell Biolabs, Inc. Santiago, USA) coated with Matrigel using serum-free medium. In the bottom chamber, serum-containing medium was used as a chemoattractant. After incubating at 37 °C for 48 h, the noninvasive cells in the top chambers were removed and the invaded cells on the lower membrane surface were fixed with 100% methanol, stained with DAPI (Beyotime Institute of Biotechnology, Haimen, China),and counted under a microscope.

The article "The circular RNA 001971/miR-29c-3p axis modulates colorectal cancer growth, metastasis, and angiogenesis through VEGFA" was retracted in 2022. Reason: lack of ethics approval or compliance.

### Expression levels determined by polymerase chain reaction (PCR)-based analysis

For miRNA, circRNA and mRNA expression determination, we extracted total RNA using TRIzol reagent (Invitrogen) following the manufacturer’s instructions. For miRNA expression determination, reverse transcription was conducted using miRNA-specific primers and a miScript Reverse Transcription kit (Qiagen, Germany) taking RNU6B expression as an endogenous control. For mRNA expression determination, SYBR green PCR Master Mix (Qiagen) was used, using GAPDH expression as an endogenous control. For circRNA expression determination, the total RNA was digested by Ribonuclease R (Epicentre, USA), and then the RNA was reverse transcribed and subjected to RT-PCR using SYBR green PCR Master Mix (Qiagen). RT-PCR assays with divergent or convergent primers were used for circRNA identification (Fig. S1). The relative fold-change was calculated by the 2^−ΔΔCT^ method. The primer sequences are listed in Table S1.

### Tumorigenicity assay in mice

Six BALB/c nude male mice (4 weeks old) were used in the experiments. All animals were randomly assigned into two groups. SW620 cells, infected with Lv-sh-NC or Lv-sh-circ-001971 (GeneChem, China) were suspended in 200 μL growth medium/Matrigel and hypodermically injected into the left axillaries of mice in the different groups. Twenty-five days after the injection, mice were sacrificed under anesthesia. The length (L) and width (W) of the tumors were measured and the tumor volumes (V) were calculated following the formula V  =  L  ×  W^2^/2 every 5 days for 25 days. At the end of the animal experiments, the tumor weights in the two groups were determined.

### Protein levels determined by immunoblotting

RIPA buffer (Sigma-Aldrich, St. Louis, MO, USA) was used to lyse the target cells and a complete protease inhibitor cocktail (Roche, USA) was used for total protein collection. Then, total proteins were separated using SDS-PAGE and transferred onto PVDF membranes. The antibodies listed below were used to incubate the blots at 4 °C overnight: anti-VEGFA (ab1316) and anti-GAPDH (ab8245, Abcam). The membranes were then incubated with an HRP-conjugated secondary antibody (1:5000). Signals were visualized using ECL (enhanced chemiluminescence) substrates (Millipore, USA) using endogenous GAPDH levels for normalization.

The article "The circular RNA 001971/miR-29c-3p axis modulates colorectal cancer growth, metastasis, and angiogenesis through VEGFA" was retracted in 2022. Reason: lack of ethics approval or compliance.

### Luciferase reporter assay

For miR-29c-3p binding to circ-001971 or the 3’UTR of VEGFA, the fragment of circ-001971 or the 3’UTR of VEGFA was amplified by PCR and cloned downstream of the Renilla gene in the psiCHECK-2 vector (Promega, Madison, WI, USA), which was named wt-circ-001971 or wt-VEGFA 3’UTR. To generate the circ-001971, VEGFA 3’UTR mutant reporters, the seed region of the circ-001971 and the VEGFA 3’UTR were mutated to remove the complementarity to miR-29c-3p, and the resulting constructs were named mut-circ-001971 and mut-VEGFA 3’UTR. HEK293 cells (ATCC, USA) were seeded into a 24-well plate. Then, HEK293 cells were cultured overnight and cotransfected with a luciferase reporter vector and miR-29c-3p mimics/inhibitor. After 48 h, the alterations in the luciferase activity were evaluated by the Dual-Luciferase Reporter Assay System (Promega) using firefly luciferase activity for normalization.

### RNA immunoprecipitation (RIP)

RIP assay was conducted to validate the predicted binding. A Magna RIP RNA-Binding Protein Immunoprecipitation Kit (17–700; Millipore, Burlington, MA, USA) according to the product’s instructions. The immunoprecipitated RNAs were reverse transcribed and subjected to RT-PCR using the PrimeScript™ RT reagent Kit (Takara, Japan) and SYBR Green PCR Master Mix (Qiagen). miR-29c-3p, circ-001971, and VEGFA levels in the immunoprecipitates were detected using specific primers.

### Statistical analysis

Each experiment was repeated at least three times. Data were processed by SPSS 17.0 and presented as the mean ± S.D. Differences between two groups were compared using Student’s *t*-test; differences among more than two groups were compared using one-way ANOVA following Turkey’s test. Pearson Correlation analysis was used to determine the relationships among miR-29c, circ-001971 and VEGFA. Kaplan-Meier analysis of overall survival by the log-rank test was used for overall survival analysis. Receiver operating characteristic (ROC) curve analysis was performed to evaluate the diagnostic and prognostic sensitivity and specificity of circ-001971 for CRC. *P < 0.05; **P < 0.01.

## Results

### Selection of circ-001971

Tissue samples were collected and verified by H&E staining (Fig. 1a). To identify circRNAs that might be related to CRC carcinogenesis, the top 11 upregulated circRNAs previously reported to be highly expressed in CRC tumor tissue samples compared with normal mucosa tissue samples (Table S2) [37], were selected for real-time PCR confirmation. Figure 1b shows that in 13 paired tumor and noncancerous tissue specimens, circ-002739, circ-001971 and circ-004028 were significantly upregulated in tumor tissues, and circ-001971 was the most upregulated (Fig. 1b). Thus, circ-001971 was selected for further experiments.

The article "The circular RNA 001971/miR-29c-3p axis modulates colorectal cancer growth, metastasis, and angiogenesis through VEGFA" was retracted in 2022. Reason: lack of ethics approval or compliance.

**Fig. 1:** Selection of circ-001971 (**a**) Pathological characteristics of the tumor and non-cancerous tissues revealed by H&E staining. **b** The expression of the top 11 upregulated circRNAs reported by the previous study was verified in 13 paired tumor and noncancerous tissues using real-time PCR. The data are presented as the mean ± SD of three independent experiments. *P < 0.05, **P < 0.01. **c** The expression of circ-001971 was examined in 70 paired tumor and noncancerous tissues using real-time PCR. **d** Circ-001971 expression was analyzed according to the TNM stage. **e** ROC curve of circ-001971 to distinguish colorectal cancer (CRC) from controls. **f** Colorectal cancer (CRC) cases were divided into two groups according to circ-001971 expression. Overall survival was analyzed by Kaplan-Meier overall survival analysis using the log-rank test. **g** ROC curve of circ-001971 to assess the diagnostic sensitivity and specificity of circ-001971 for CRC

In 70 paired tissue specimens, circ-001971 expression was significantly upregulated, consistent with the previous small sample size examination (Fig. 1c). Next, we analyzed circ-001971 expression according to the TNM stage and found that circ-001971 expression was higher in specimens at advanced TNM stages (III + IV) than in specimens at early stages (I + II; Fig. 1d). To further validate the effect of circ-001971 on CRC, the association between the expression of circ-001971 and the clinical indicators of CRC patients was detected. Seventy cases were assigned into two groups, high and low circ-001971 expression groups, by the median value of circ-001971 expression. Table 1 shows that high circ-001971 expression was dramatically related to advanced TNM stages and lymphatic metastasis. Moreover, we employed a Cox proportional hazards regression model to detect the overall survival rate and pathologic features of the 70 CRC patients. Univariate analysis revealed that the TNM stage, lymph node metastasis and circ-001971 expression caused remarkable differences in the overall survival rate. Mutivariable analysis demonstrated that the TNM stage and circ 001971 expression led to the differences in overall survival rate with statistical significance (Table 2). To determine circ-001971 as a biomarker of CRC, we performed ROC curve analysis to evaluate the diagnostic (Fig. 1e) and prognostic (Fig. 1g) sensitivity and specificity of circ-001971 for CRC. The area under the curve was 0.788 (Fig. 1e) or 0.792 (Fig. 1g), which shows that circ-001971 has a potential diagnostic and prognostic capability (Fig. 1e and g). Kaplan-Meier curves of overall survival by log-rank test demonstrated that the overall survival rate of patients in the low circ-001971 expression group was higher (Fig. 1f), suggesting the underlying effect of circ-001971 on CRC.

The article "The circular RNA 001971/miR-29c-3p axis modulates colorectal cancer growth, metastasis, and angiogenesis through VEGFA" was retracted in 2022. Reason: lack of ethics approval or compliance.

### The effects of circ-001971 on the proliferation and invasion of CRC cells and the angiogenesis of HUVECs

To investigate the specific functions of circ-001971 in CRC carcinogenesis, we examined its expression in five CRC cell lines (HT29, HCT116, LoVo, SW480, and SW620) and a normal cell line, FHC. Consistent with its expression in tissues, the expression of circ-001971 was significantly increased within CRC cells compared with FHC cell lines (Fig. 2a) and was more highly increased in HCT116 and SW620 cells (Fig. 2a). We transfected si-circ-001971#1 and si-circ-001971#2 to conduct circ-001971 knockdown in HCT116 and SW620 cells, and performed real-time PCR to verify the transfection efficiency. Then, we selected si-circ-001971#1 as the siRNA targeting circ-001971 because of its greater efficiency (Fig. 2b).

**Fig. 2:** The effect of circ-001971 on CRC cell invasion and HUVEC tube formation (**a**) The expression of circ-001971 in five CRC cell lines, HT29, HCT116, LoVo, SW480, and SW620, and a normal cell line was examined using real-time PCR. **b** The knockdown of circ-001971 was achieved in HCT116 and SW620 cells by transfection with si-circ-001971#1 or si-circ-001971#2, as confirmed using real-time PCR. (C-E) HCT116 and SW620 cells were transfected with si-circ-001971 and examined for DNA synthesis (**c**) and cell proliferation (**d-e**). **f-g** HCT116 and SW620 cells were transfected with si-circ-001971 and examined for cell invasion using Transwell assays. **h-i** We collected conditioned medium from circ-001971-knockdown or control SW620 cells (si-circ-001971 CM and si-NC CM), cultured HUVECs in these two CM samples, and examined for the tube formation capacity. The data are presented as the mean ± SD of three independent experiments. *P < 0.05, **P < 0.01, compared to FHC cells or the si-NC group

Next, we transfected HCT116 and SW620 cell lines with si-circ-001971 and determined the proliferation and invasion of cells. After knocking down circ-001971, the DNA synthesis capacity (Fig. 2c), cell viability (Fig. 2d-e), and cell invasion (Fig. 2f-g) were all significantly inhibited. To further investigate the effects of circ-001971 on HUVEC tube formation through the tumor microenvironment, we collected conditioned medium from circ-001971-knockdown or control SW620 cells (si-circ-001971 CM and si-NC CM), cultured HUVECs in these two CM, respectively, and examined HUVEC angiogenesis in different CM. Figure 2h-i shows that culture with si-circ-001971 CM significantly suppressed HUVEC tube formation compared with culture in si-NC CM.

The article "The circular RNA 001971/miR-29c-3p axis modulates colorectal cancer growth, metastasis, and angiogenesis through VEGFA" was retracted in 2022. Reason: lack of ethics approval or compliance.

### Effects of circ-001971 on CRC growth in vivo

To further confirm the tumor suppressor roles of circ-001971 knockdown, we constructed lentivirus containing shRNA targeting circ-001971 (Lv-sh-circ-001971) and performed real-time PCR to verify the knockdown efficiency (Fig. 3a). Next, six animals were randomly assigned into two groups (*n* = 3), and SW620 cells infected with Lv-sh-NC (negative control) or Lv-sh-circ-001971, were hypodermically injected into the left axillaries of the mice in these two groups (Fig. 3b). As shown in Fig. 3c and d, circ-001971 knockdown significantly reduced the tumor volumes at every measurement time point and reduced the tumor weight determined at the end of the experiment. These data indicate that circ-001971 knockdown inhibits CRC tumor growth in vivo.

**Fig. 3:** Effects of circ-001971 on CRC growth in vivo (**a**) Lentivirus containing shRNA targeting circ-001971 was constructed and the knockdown efficiency was verified by real-time PCR. **b** Six animals were randomly assigned into two groups (*n* = 3). SW620 cells infected with Lv-sh-NC or Lv-sh-circ-001971 were hypodermically injected into the left axillaries of mice in different groups. Twenty-five days after the injection, when the diameters of the resulting tumors measured approximately 5 mm, the rats were sacrificed under anesthesia. **c** The length (L) and width (W) of the tumors were measured with calipers every 5 days for 25 days and the tumor volumes were calculated. **d** At the end of the animal experiments, all the animals were sacrificed under anesthesia, and the tumor weight was determined. **P < 0.01, compared to Lv-sh-NC group

### Selection and verification of miRNAs related to circ-001971 and CRC angiogenesis

CircRNAs act as miRNA sponges to offset miRNA-induced inhibition of downstream target genes [38]. To investigate the molecular mechanism of circ-001971 functioning in CRC growth and metastasis, we screened for miRNAs that may be related to CRC metastasis and may target VEGFA, a key regulator of tumor angiogenesis [39]. According to the online microarray expression profile GSE126093, a total of 440 miRNAs were upregulated and 74 were down-regulated in CRC tissue samples than that within normal control tissue samples (*p* < 0.05, │logFC│ > 0.6) (Fig. 4a). In circ-001971 knocked-down HCT116 and SW620 cells, the protein levels of VEGFA were also significantly decreased (Fig. 4b-c), suggesting the potential crosstalk between circ-001971 and VEGFA. Next, we employed TargetScan to predict miRNAs that might target VEGFA. Among the 627 predicted miRNAs, 16 miRNAs were down-regulated in CRC reported by GSE126093. Among the 16 miRNAs, 3 were predicted to target circ-001971, namely, miR-29c-3p, miR-497-5p, and miR-943 (Fig. 4d).

The article "The circular RNA 001971/miR-29c-3p axis modulates colorectal cancer growth, metastasis, and angiogenesis through VEGFA" was retracted in 2022. Reason: lack of ethics approval or compliance.

**Fig. 4:** Selection and verification of miRNAs related to circ-001971 and CRC angiogenesis (**a**) Upregulated and downregulated miRNAs in CRC tissues compared to that in noncancerous tissues according to the online microarray expression profile GSE126093. **b-c** HCT116 and SW620 cells were transfected with si-circ-001971, and the protein levels of VEGFA were examined by immunoblotting. (**d**) TargetScan was used to predict miRNAs that might target VEGFA. Among the 627 predicted miRNAs, 16 miRNAs were downregulated miRNAs in CRC, as reported by GSE126093. Among the 16 miRNAs, 3 were predicted to target circ-001971, including miR-29c-3p, miR-497-5p, and miR-943. **e** Overexpression of the three candidate miRNAs was conducted in HCT116 and SW620 cells by the transfection with miRNA mimics. The transfection efficiency was confirmed by real-time PCR. Then, HCT116 and SW620 cells were transfected by miRNA mimics and examined for (**f**) the expression of circ-001971 by real-time PCR and (**g**) the expression of VEGFA by real-time PCR. miR-29c-3p was selected for further experiments. **h** miR-29c-3p inhibition was conducted in HCT116 and SW620 cells by the transfection of miR-29c-3p inhibitor. The transfection efficiency was verified by real-time PCR. **i** HCT116 and SW620 cells were transfected with miR-29c-3p inhibitor and the expression of circ-001971 was examined by real-time PCR. **j** HCT116 and SW620 cells were transfected by si-circ-001971 and examined for the expression of miR-29c-3p by real-time PCR. (K-L) HCT116 and SW620 cells were transfected with miR-29c-3p mimics or inhibitor, and the protein levels of VEGFA were by immunoblotting. *P < 0.05; **P < 0.01, compared to si-NC, mimics-NC or inhibitor NC group

To further confirm the miRNA that might mediate the crosstalk between circ-001971 and VEGFA, we transfected miRNA mimics to overexpress the three candidate miRNAs in HCT116 and SW620 cells, and performed real-time PCR to verify the transfection efficiency (Fig. 4e). Next, we transfected HCT116 and SW620 cell lines with miRNA mimics and examined the expression of circ-001971 and VEGFA. As shown in Fig. 4f and g, all three miRNAs inhibited the expression of VEGFA within both CRC cells, however, only miR-29-3p strongly inhibited circ-001971 expression within both CRC cell lines. Thus, we selected miR-29c-3p for further experiments.

We transfected miR-29c-3p inhibitor to conduct miR-29c-3p inhibition within HCT116 and SW620 cell lines, as confirmed by real-time PCR (Fig. 4h). In miR-29c-3p inhibited HCT116 and SW620 cells, circ-001971 expression was significantly upregulated (Fig. 4i); in circ-001971 knockdown HCT116 and SW620 cell lines, miR-29c-3p expression was dramatically upregulated (Fig. 4j). Moreover, within HCT116 and SW620 cell lines, miR-29c-3p overexpression dramatically decreased, while miR-29c-3p inhibition increased VEGFA protein levels (Fig. 4k-l).

The article "The circular RNA 001971/miR-29c-3p axis modulates colorectal cancer growth, metastasis, and angiogenesis through VEGFA" was retracted in 2022. Reason: lack of ethics approval or compliance.

### miR-29c-3p directly binds to circ-001971 and VEGFA

To investigate the putative miR-29c-3p binding to circ-001971 and VEGFA, we performed luciferase reporter and RIP assays. We constructed two kinds of reporter vectors, wild-type and mutant, which named wt-circ-001971/mut-circ-001971 and wt-VEGFA 3’UTR/mut-VEGFA 3’UTR, respectively. In the mutant reporter vectors, 4 bases were mutated in the predicted miR-29c-3p binding site of (Fig. 5a and c). Next, we cotransfected HEK293 cells with these vectors and miR-29c-3p mimics/inhibitor, and determined the luciferase activity. Wild-type vector (wt-circ-001971 and wt-VEGFA 3’UTR) luciferase activity was dramatically reduced via the overexpression of miR-29c-3p, and it was increased via the inhibition of miR-29c-3p. Once the putative binding site was mutated, the luciferase activity was reduced to almost the original value (Fig. 5b and d). To further confirm the binding, RIP assays were performed. Based on the results, circ-001971, VEGFA and miR-29c-3p were associated with AGO2; in RNA extracted from the protein precipitate, circ-001971, VEGFA and miR-29c-3p levels were twice as high as those in the IgG sample (Fig. 5e). Moreover, endogenous circ-001971 and VEGFA pull-down by AGO2 was enriched after miR-29c-3p overexpression (Fig. 5f). These data confirmed that circ-001971 and VEGFAbind to miR-29c-3p in a AGO2-associated manner.

**Fig. 5:** miR-29c-3p directly binds to circ-001971 and VEGFA (**a-b**) Two different types of luciferase reporter vectors were constructed: wild-type circ-001971 and VEGFA 3’UTR, and mutant-type circ-001971 and VEGFA 3’UTR; mutant-type vectors contained a 4 bp mutation in the predicted miR-29c-3p binding site. **c-d** The above vectors were cotransfected into HEK293 cells with miR-29c-3p mimics or miR-29c-3p inhibitor and examined for luciferase activity. **e** RIP assays were performed to confirm the binding of miR-29c-3p to circ-001971 and VEGFA using an AGO2 antibody. The levels of miR-29c-3p, circ-001971 and VEGFA in precipitated AGO2 proteins were examined using real-time PCR. **f** Endogenous circ-001971 and VEGFA 3’UTR pull-down by AGO2 upon overexpression of miR-29c-3p was determined using RIP assays. The data are presented as the mean ± SD of three independent experiments. **P < 0.01, compared to mimics-NC, inhibitor-NC, IgG group

The article "The circular RNA 001971/miR-29c-3p axis modulates colorectal cancer growth, metastasis, and angiogenesis through VEGFA" was retracted in 2022. Reason: lack of ethics approval or compliance.

### The circ-001971/miR-29c-3p axis modulates the tube formation capacity of HUVECs

After confirming circ-001971 binding to miR-29c-3p, the study continued to investigate the dynamic effects of circ-001971 and miR-29c-3p on HUVEC tube formation. First, HCT116 and SW620 cells were cotransfected with miR-29c-3p inhibitor and si-circ-001971, and the protein levels of VEGFA were examed. As shown in Fig. 6a-b, in both cell lines, miR-29c-3p inhibition increased, while circ-001971 knockdown decreased the protein levels of VEGFA, and the effects of circ-001971 knockdown on VEGFA protein levels were significantly reversed by miR-29c-3p inhibition. Then, different CM samples were collected for HUVEC culture. As shown in Fig. 6c-d, miR-29c-3p inhibition significantly enhanced, while circ-001971 knockdown inhibited the tube formation ability of HUVECs and the effects of circ-001971 knockdown on HUVEC tube formation were significantly reversed by miR-29c-3p inhibition. Overall, these data indicate that the circ-001971/miR-29c-3p axis could modulate VEGFA protein levels and HUVEC tube formation.

**Fig. 6:** The circ-001971/miR-29c-3p axis modulates the tube formation capacity of HUVECs (**a-b**) HCT116 and SW620 cells were cotransfected with miR-29c-3p inhibitor and si-circ-001971, and the protein levels of VEGFA were determined. **c-d** HUVECs were cultured in miR-29c-3p inhibitor and si-circ-001971 transfected SW620 cell conditioned medium (CM) and assayed for tube formation capacity. *P < 0.05, **P < 0.01, compared to si-NC + inhibitor-NC group; ##*P* < 0.01, compared to si-circ-001971 + inhibitor-NC group

### miR-29c-3p and VEGFA expression in tissue samples and their correlation with circ-001971

As a further confirmation, we performed real-time PCR to examine miR-29c-3p and VEGFA expression in tissue samples. Figure 7a-b shows that the expression of miR-29c-3p was obviously inhibited while the expression of VEGFA was enhanced within tumor tissues compared with non-cancerous tissue samples. Consistent results were revealed obtained by IHC and immunoblotting assays that VEGFA protein contents within tumor tissue samples showed to be increased as compared to those within non-cancerous tissue samples (Fig. 7c-d). In addition, miR-29c-3p was negatively related to circ-001971 and VEGFA (Fig. 7e-f); circ-001971 was positively related to VEGFA (Fig. 7g).

**Fig. 7:** Expression of miR-29c-3p, HIF1α and VEGFA in tissue specimens and their correlation with circ-001971 (**a-b**) Expression of VEGFA and miR-29c-3p in 70 paired tumor and noncancerous tissue samples was examined using real-time PCR. **c** VEGFA contents in tumor and noncancerous tissues were examined using IHC assays. **d** VEGFA protein levels in tumor and non-cancerous tissues were examined using immunoblotting. **e-g** The correlation of circ-001971, miR-29c-3p, and VEGFA was analyzed using Pearson’s correlation analysis. *P < 0.05, compared to noncancerous tissue samples

The article "The circular RNA 001971/miR-29c-3p axis modulates colorectal cancer growth, metastasis, and angiogenesis through VEGFA" was retracted in 2022. Reason: lack of ethics approval or compliance.

## Discussion

Herein, we demonstrate that the circ-001971/miR-29c-3p axis modulates CRC cell proliferation and invasion ability and HUVEC angiogenesis by targeting VEGFA. In rats bearing SW620 cell-derived tumors, circ-001971 knockdown significantly inhibited tumor growth compared to the control group. In tumor tissues, circ-001971 and VEGFA expression was significantly increased whereas miR-29c-3p expression was reduced, further suggesting that circ-001971 counteracts miR-29c-3p-induced inhibition of VEGFA by acting as a ceRNA, therefore aggravating CRC growth, metastasis, and angiogenesis.

The dysregulation of ncRNAs in CRC has been widely reported. Xiong et al. reported that 2662 lncRNAs and 2398 mRNAs in total were differentially expressed in 5-FU-based chemoradiation resistant HCT116 cells. By using KEGG (Kyoto Encyclopedia of Genes and Genomes) pathway analysis, they observed that the related signaling pathways, including the JAK-STAT, PI3K-Akt and NF-kappa B signaling pathways, were involved in CRC progression [40]. Moreover, miRNA-mRNA crosstalk and its effects on CRC have been widely studied [41], whereby each CRC metastatic process, consisting of new blood vessel formation, invasion, intravascular perfusion, circulation, extravasation, and metastatic colonization could be impacted by these miRNAs [42]. Unlike these two kinds of ncRNAs, the role and mechanism of circRNAs in CRC need further investigation. According to Bachmayr et al. [43], we selected the 11 circRNAs that were most upregulated in CRC tissues for further investigation. Of them, circ-001971 expression was more upregulated in 13 CRC tissue specimens. Interestingly, circ-001971 expression was higher in specimens in advanced TNM stages, and high circ-001971 expression was significantly related to CRC patient adverse prognosis, indicative of the underlying effect of circ-001971 on CRC progression.

Tumor growth would be limited when tumors grow beyond 2–3 mm^3^ in size because of the lack of vasculature [44]. In this case, the angiogenic switch would be triggered for survival, and cancer cell invasion and metastasis would be promoted. Herein, circ-001971 knockdown significantly inhibited CRC cell proliferation and invasion and HUVEC angiogenesis, suggesting that circ-001971 may have a strong impact on CRC progression. As further evidence, in rats bearing SW620 cell-derived tumors, knocking down circ-001971 significantly inhibited the growth of tumors, indicating that circ-001971 knockdown exerts a tumor-suppressive effect.

The article "The circular RNA 001971/miR-29c-3p axis modulates colorectal cancer growth, metastasis, and angiogenesis through VEGFA" was retracted in 2022. Reason: lack of ethics approval or compliance.

Regarding the molecular mechanism, circRNAs usually function by acting as miRNA sponges. One of the mechanisms by which hsa_circ-001569 enhanced the expression of the miR-145 functional targets E2F5, BAG4 and FMNL2 is by acting serving as a miR-145 sponge, while promoting the capacity of CRC cells to proliferate and invade [45]. Hsa_circ-0020397 inhibited the miR-138 activity on its downstream targets including TERT (telomerase reverse transcriptase) and PD-L1 (programmed death-ligand 1), and thus antagonized miR-138 suppression of CRC cell growth [46]. In the present study, miRNAs that may be related to CRC metastasis and may simultaneously target circ-001971 and VEGFA were selected. Of the three identified miRNAs, miR-29c-3p overexpression inhibited circ-001971 expression more than miR-497-5p and miR-943 did. Consistent with previously-reported circRNA-miRNA pairs, circ-001971 and miR-29c-3p negatively regulated each other. More importantly, miR-29c-3p negatively modulated the protein levels of VEGFA, suggesting that circ-001971 may exert its effect on CRC proliferation, invasion, and angiogenesis through miR-29c-3p.

As further evidence of online target prediction tools indicated that miR-29c-3p could directly target both circ-001971 and VEGFA. It has been revealed that miR-29c-3p serves as an antitumor miRNA in a number of cancers and its expression is downregulated in cancers including head and neck cancers [47], endometrial carcinoma [48], gastric cancer [49], and colorectal cancer [50]. Has-miR-29c-3p overexpression was shown to decrease the capacity of CRC cells to proliferate and migrate [50]. In the present study, consistent with the negative dual-regulation of circ-001971 and miR-29c-3p, HUVEC angiogenesis was remarkably attenuated via circ-001971 knockdown but enhanced via the inhibition of miR-29c-3p, while the inhibition of miR-29c-3p significantly attenuated the effect of circ-001971 knockdown. In addition, circ-001971/miR-29c-3p axis also modulated VEGFA protein levels. As we have mentioned, VEGFA expression is considered to be one of the most critical proangiogenic factors for tumor cell secretion [11, 12]. Herein, abnormally increased VEGFA protein levels in CRC cells were observed. Moreover, VEGFA protein levels could be dramatically decreased by circ-001971 silencing but enhanced via miR-29c-3p inhibition. In summary, miR-29c-3p and upstream circ-001971 exert their functions on CRC proliferation, invasion, and angiogenesis through VEGFA.

The article "The circular RNA 001971/miR-29c-3p axis modulates colorectal cancer growth, metastasis, and angiogenesis through VEGFA" was retracted in 2022. Reason: lack of ethics approval or compliance.

## Conclusions

As further evidence of the above findings, the expression of VEGFA was upregulated, whereas the expression of miR-29c-3p was downregulated in tumor tissue samples. miR-29c-3p was negatively correlated with circ-001971 and VEGFA, while circ-001971 was positively correlated with VEGFA. Overall, the circ-001971/miR-29c-3p axis modulates CRC proliferation, invasion, and angiogenesis through VEGFA. We provide a new rationale for the effect of the circRNA-miRNA-mRNA network on CRC progression.

## Supplementary information

**Additional file 1: Fig. S1.** Identification of circ-001971. (A) RT-PCR assay with divergent or convergent primers indicating the existence of circ-001971 in SW620 cells. GAPDH was used as a negative control. cDNA: complementary DNA. gDNA: genomic DNA. (C) qRT-PCR analysis of the expression of circRNA-001971 after RNase R treatment in SW620 cells. **P < 0.01, compared to RNase R^−^ group.

**Additional file 2: Table S1.** the sequence of primers.

**Additional file 3: Table S2**. The top 11 upregulated circular RNA in CRC tumor tissue samples than normal mucosa tissue samples.

## Data Availability

Not applicable.

## Abbreviations

CM: condition media
ceRNAs: Competing endogenous RNAs
circRNAs: Circular RNAs
CRC: Colorectal cancer
H&E: Hematoxylin and eosin
IHC: Immunohistochemical
KEGG: Kyoto Encyclopedia of Genes and Genomes
lncRNAs: Long non-coding RNAs
ncRNAs: Non-coding RNAs
miRNAs: micrornas
PD-L1: Programmed death-ligand 1
ROC: Receiver operating characteristic
TERT: Telomerase reverse transcriptase
VEGFA: Vascular endothelial growth factor A
